# Extra-axonal restricted diffusion as an in-vivo marker of reactive microglia

**DOI:** 10.1038/s41598-019-50432-5

**Published:** 2019-09-25

**Authors:** Maxime Taquet, Aleksandar Jankovski, Gaëtan Rensonnet, Damien Jacobs, Anne des Rieux, Benoît Macq, Simon K. Warfield, Benoît Scherrer

**Affiliations:** 1 Computational Radiology Laboratory, Boston Children’s Hospital, Harvard Medical School, Boston, USA; 2 Department of Neurology, Boston Children’s Hospital, Harvard Medical School, Boston, USA; 3 ICTEAM Institute, Université catholique de Louvain, Louvain-la-Neuve, Belgium; 4 Department of Psychiatry, University of Oxford, Oxford, United Kingdom; 5 Institute of Neuroscience, Université catholique de Louvain, Louvain-la-Neuve, Belgium; 6 Department of Neurosurgery, Université catholique de Louvain, CHU UCL Namur, Yvoir, Belgium; 7 Ecole Polytechnique Fédérale de Lausanne, Lausanne, Switzerland; 8 Louvain Drug Research Institute, Université catholique de Louvain, Woluwe-Saint-Lambert, Belgium

**Keywords:** Diseases of the nervous system, Diagnostic markers

## Abstract

Reactive microgliosis is an important pathological component of neuroinflammation and has been implicated in a wide range of brain diseases including brain tumors, multiple sclerosis, Parkinson’s disease, Alzheimer’s disease, and schizophrenia. Mapping reactive microglia *in-vivo* is often performed with PET scanning whose resolution, cost, and availability prevent its widespread use. The advent of diffusion compartment imaging (DCI) to probe tissue microstructure *in vivo* holds promise to map reactive microglia using MRI scanners. But this potential has never been demonstrated. In this paper, we performed longitudinal DCI in rats that underwent dorsal root axotomy triggering Wallerian degeneration of axons—a pathological process which reliably activates microglia. After the last DCI at 51 days, rats were sacrificed and histology with Iba-1 immunostaining for microglia was performed. The fraction of extra-axonal restricted diffusion from DCI was found to follow the expected temporal dynamics of reactive microgliosis. Furthermore, a strong and significant correlation between this parameter and histological measurement of microglial density was observed. These findings strongly suggest that extra-axonal restricted diffusion is an *in-vivo* marker of reactive microglia. They pave the way for MRI-based microglial mapping which may be important to characterize the pathogenesis of neurological and psychiatric diseases.

## Introduction

The presence of reactive microglia in neuroinflammation is thought to play a key role in the pathogenesis of a range of brain diseases such as Alzheimer’s disease^1^, Parkinson’s disease^2^, multiple sclerosis^3^, depression^4^, and schizophrenia^5^ among others. More generally, neuroinflammation is an increasingly recognized important pathological pathway in a variety of psychiatric disorders and has become a promising target for treatment^6,7^. Reactive microgliosis also has a pivotal role in the pathogenesis of brain tumors such as glioblastomas wherein tumor cells attract and then activate microglia^8^.

The ability to effectively and efficiently map the presence and status of microglial cells *in vivo* is therefore becoming increasingly important to investigate the pathogenesis of brain diseases and to assess response to treatment. To avoid the invasiveness and sparsity of biopsies, investigators have relied on positron emission tomography (PET) with specific ligands to map reactive microglia^2^. However, the cost and availability of PET scanning prevent its widespread use and its limited resolution precludes the identification of neuroinflammatory loci or specific inflamed brain circuits.

A promising alternative to PET scans to map reactive microglia is the use of diffusion compartment imaging (DCI)^9,10^—a novel approach based on diffusion-weighted magnetic resonance imaging (DW-MRI) to image the microstructure of neural tissues. Unlike diffusion tensor imaging (DTI), DCI considers that there are multiple microstructural environments in each voxel and provides a separate parameterization for the signal arising from each of them^11^. The ability of DCI to detect glial cells has been theoretically suggested^12,13^ but has never been demonstrated.

A reliable empirical setup to investigate reactive microglia mapping is to trigger Wallerian degeneration in the spinal cord of rats^14^. Wallerian degeneration is the pathological process that occurs following axonal injury and includes axonal loss, myelin clearance, and the recruitment of reactive microglia. Its temporal evolution is well established^14^ and a wealth of studies have demonstrated the sensitivity of DTI to axonal loss and myelin clearance^15–21^. The consensus that emerges from these studies is that radial diffusivity starts increasing weeks after injury and is a marker of myelin clearance, while axial diffusivity decreases in the acute phase before normalization and is a marker of axonal loss. DTI studies however have failed to map reactive microglia.

In this study, we used DIAMOND^10^, a recently developed DCI model, to longitudinally characterize the tissue microstructure of seven rats (3 control and 4 injured) imaged at baseline, and at 4, 13, 37, and 51 days after unilateral dorsal root axotomy (or a sham intervention). After 51 days, rats were sacrificed and we compared the last DIAMOND parameters to histological measurements of microglial density. The two-compartment DIAMOND model used has one compartment that captures the axonal signal (represented by parameters that have their DTI counterpart) and one compartment that captures the extra-axonal restricted diffusion thought to arise from reactive microglia.

## Results

This section first presents the histological validation of the pathological features occurring in our experimental setup. Next, the temporal and spatial evolutions of DIAMOND parameters are presented. Finally, the correlation between the fraction of extra-axonal restricted diffusion (*f*_ear_) of DIAMOND and histological microglial density are presented.

### Histological validation of pathological features

SMI-312 staining (Fig. 1A) exhibits a markedly significantly lower axonal density on the ipsilateral than on the contralateral side (decrease by over 60%; two-sample t-test $t(30)=4.60$, $p=3.6\times {10}^{-5}$) and on the ipsilateral side than in control rats (decrease by over 60%; two-sample t-test $t(26)=5.06$, $p=1.4\times {10}^{-5}$) but no significant difference was observed between control rats and the contralateral side of injured rats (two-sample t-test $t(26)=0.48$, $p=0.32$). This provides evidence for axonal degeneration on the ipsilateral side but not on the contralateral side.

**Figure 1:** Histological validation of the animal model of injury 51 days rhizotomy. (**A**) SMI-312 staining is used to mark neurofilament loss and demonstrates that neurofilament density is significantly lower on the side of lesion (ipsilateral). (**B**) Iba-1 staining is used to mark reactive microglia and demonstrates that microglial density is significantly higher on the side of the lesion. (**C**) LFB staining is used to mark the myelin and demonstrates that myelin intensity is significantly lower on the side of the lesion. The absence of significant differences for all three stainings between the contralateral side and the control rats indicates that the contralateral side can be reliably used as control in longitudinal analyses. Scale bars are 100 *μ*m. Error bars indicate ±1 standard error. *p < 0.05, **p < 0.005, ***p < 0.0005.

Iba-1 staining (Fig. 1B) exhibits significantly higher microglial density on the ipsilateral than on the contralateral side (six-fold increase; two-sample t-test $t(26)=4.81$, $p=2.7\times {10}^{-5}$) and on the ipsilateral side than in control rats (six-fold increase; two-sample t-test $t(30)=3.65$, $p=4.9\times {10}^{-4}$) but no significant difference was observed between control rats and the contralateral side of injured rats (two-sample t-test $t(26)=0.19$, $p=0.42$). This provides evidence for the presence of reactive microglia on the ipsilateral side.

The intensity of LFB staining (Fig. 1A) was significantly lower on the ipsilateral side than on the contralateral side (decrease by approximately 50%; two-sample t-test $t(30)=2.19$, $p=0.018$) and on the ipsilateral side than in control rats (decrease by approximately 50%; two-sample t-test $t(26)=4.14$, $p=1.6\times {10}^{-4}$) but no significant difference was observed between control rats and the contralateral side of injured rats (two-sample t-test $t(26)=0.58$, $p=0.28$). This provides evidence for myelin loss on the ipsilateral side.

These results confirm the validity of the rhizotomy model by demonstrating the known pathological features of the Wallerian degeneration. They also confirm the preservation of the contralateral dorsal column which has microstructural properties similar to control rats so that they can be used as a control for the rest of the analyses.

### Temporal evolution of DIAMOND parameters

An example of maps of all DIAMOND parameters and their evolution with time for one injured rat at a location in the spinal cord rostral to the lesion, between L2 and T12 is depicted in Fig. 2. The temporal evolution of DIAMOND parameters reveals four main findings (Fig. 3 and Table 1).

**Figure 2:** DIAMOND parameters and their evolution through time for one injured rat. The DIAMOND parameters include the fascicular axial (*λ*_‖_) and radial (*λ*_⊥_) diffusivities, and the fraction (*f*_ear_) and diffusivity (*d*_ear_) of the extra-axonal restricted compartment. The displayed axial slice has been selected between the lesion and the most rostral aspect of the region of interest. Grey matter has been masked out. The insets represent the dorsal roots where the axotomy was performed.

**Figure 3:** Evolution of the DIAMOND parameters measured at 5 time points. (**A**) The axial diffusivity exhibits a significant decrease in the acute phase followed by a relative normalization. (**B**) The relative normalization of the axial diffusivity is dominated by the most distal (rostral) part of the axons with respect to the lesion site whereas it remains substantially lower near the lesion. (**C**) The radial diffusivity only becomes significantly higher in the late stage of Wallerian degeneration. (**D**) The heterogeneity index remains broadly unchanged throughout the process. (**E**) The extra-axonal restricted fraction (*f*_ear_) exhibits a two-stage increase. (**F**) The diffusivity in the extra-axonal restricted compartment (*d*_ear_) exhibits a two-stage decrease. All reported p-values are Bonferroni-corrected: *p < 0.05, **p < 0.005, *** *p* < 0.0005.

**Table 1:** Summary statistics (*t*-scores and *p*-values) for the temporal evolution of the DIAMOND parameters.

Property	4 days		13 days		37 days		51 days	
	*t*(30)	*p*	*t*(30)	*p*	*t*(30)	*p*	*t*(30)	*p*
*λ*_‖_	9.91	5.7 × 10^−10^	6.02	1.3 × 10^−5^	3.11	0.040	1.61	0.70
*λ*_⊥_	0.154	1.00	0.880	0.99	0.970	0.976	3.09	0.043
Hei	0.837	0.99	0.220	1.00	1.48	0.79	1.18	0.930
*f*_ear_	10.0	4.3 × 10^−10^	4.66	6.9 × 10^−4^	8.10	4.9 × 10^−8^	11.0	4.5 × 10^−11^
*d*_ear_	3.17	0.034	1.70	0.64	8.92	6.1 × 10^−9^	7.62	1.7 × 10^−7^

All p-values are Bonferroni-corrected.

First, a significant decrease in fascicular axial diffusivity is observed in the acute phase followed by a relative normalization (Fig. 3A). The relative normalization is not homogenous along the rostro-caudal axis and the white matter most caudal (proximal to the lesion) remains affected with a substantially lower fascicular axial diffusivity (*λ*_‖_) 51 days after the injury (Fig. 3B). Second, a significant increase in fascicular radial diffusivity (*λ*_⊥_) is observed in the late phase only (Fig. 3C). Third, the heterogeneity index exhibits no significant change throughout the degeneration process (Fig. 3D). Finally, the fraction (*f*_ear_) and diffusivity (*d*_ear_) of the compartment representing extra-axonal restricted diffusion follow parallel and opposite temporal evolutions (Fig. 3E,F). In the acute phase, *f*_ear_ increases and *d*_ear_ decreases. These changes are exacerbated in the late phase. At 51 days, the isotropic fraction reached a value of 0.30 which is 2.66 times higher than the baseline value while the diffusivity reached a value of 1.13 *μ*m^2^/ms which is 36% its baseline value.

These findings suggest that there are three distinct temporal processes at play: one with a mostly acute component (detected by changes in fascicle-specific *λ*_‖_), one with a mostly late component (detected by changes in fascicle-specific *λ*_⊥_), and one with both an acute component and an exacerbation in the late phase (detected by *f*_ear_ and *d*_ear_).

### Correlation between DIAMOND and histology

To test whether the fraction of extra-axonal restricted diffusion (*f*_ear_) is a marker of reactive microglia, we analyzed the correlation between *f*_ear_ extracted from DIAMOND 51 days after surgery and the microglial density extracted from histology with Iba-1 immunostaining. On the ipsilateral side, both *f*_ear_ and the microglial density increase closer to the lesion (i.e. more caudally) whereas on the contralateral side, both parameters remain broadly constant throughout the region of interest (Fig. 4A,B). A strong and significant correlation between *f*_ear_ and the microglial density was observed (Pearson correlation $r=0.94$, $p < {10}^{-6}$; Fig. 4C). An example of the correspondance between the two parameters for one rat and two vertebral levels is depicted in Fig. 4D.

**Figure 4:** Relationship between the microglial density estimated with histology at 51 days and the isotropic fraction from DIAMOND. (**A**,**B**) On the ipsilateral side, both the microglial density and the isotropic fraction decrease steadily from the site of the lesion (L2) towards the distal (rostral) part of axons (T13). On the contralateral side, both variables remain broadly constant and lower than the values on the ipsilateral side. The dashed lines connect the mean isotropic fraction while the continuous lines connect the mean glial density. (**C**) There is a strong correlation between the microglial density and the isotropic fraction. (**D**) Examples of histological slices and the corresponding isotropic fraction at two spinal levels demonstrating the larger recruitment of microglial cells near the lesion (L2) than away from it (T13). The arrows show a large density of macrophages in the dorsal root at L2 (corresponding to the stem of the lesioned rootlets) but not at T13 suggesting an active migration process near the lesion. Scale bar: 100 *μ*m.

## Discussion

The strong correlation between *f*_ear_ and microglial density observed in this study suggests that the fraction of extra-axonal restricted diffusion captures changes due to reactive microgliosis. Two other elements further support this claim. First, the time course of the changes in *f*_ear_ and *d*_ear_ are compatible with the known time course of reactive microgliosis. Histological evidence indeed demonstrates that Wallerian degeneration in the central nervous system presents reactive microglial infiltration as early as 7 days after injury at the lesion site^22^ while the peak of reactive microglial density occurs around 21 days after injury^14^. Second, the extra-axonal restricted compartment of DIAMOND (represented by an isotropic tensor whose diffusivity is estimated from the data) as used in this study has been defined specifically to capture the diffusion of water molecules trapped in closed isotropic environments such as reactive mircroglia. Unlike axons, microglial cells do not favor a particular direction of diffusion and are morphologically more isotropic^23^. The use of an isotropic tensor (as used in some studies^24,25^) rather than a closed sphere with fixed radius (as suggested in others^11,12^) for modeling this compartment is justified by the presence of microglial cells featuring a broad range of diameters. The cumulative signal arising from all these individual restricted compartments is therefore well represented by a Gaussian distribution, which leads to a tensor in our signal formula. This is analogous in DTI to the use of a cylindrical tensor rather than a cylinder to model the cumulative signal arising from a bundle of individual axons.

Importantly, what is referred to as the extra-axonal restricted compartment in the present study is different from the extracellular free-water mapping developed by Pasternak *et al*.^26^. In the latter, the diffusion coefficient of the isotropic compartment is set to the free diffusivity of water molecules at 37 °C and is meant to represent water freely diffusing in the extracellular space and the cerebrospinal fluid (CSF). In the absence of histological validation, the underpinning pathological processes leading to raised extracellular free water remains speculative. Neuroinflammation^27^ and white matter atrophy^28^ have been hypothesized. Of note, the characteristic displacement of water molecules for such a free water diffusion coefficient (*D*_0_ = 3 *μ*m^2^/ms) with common values of the effective diffusion time (${\tau }_{{\rm{eff}}}\sim 100\,{\rm{ms}}$) is of the order of 40 *μm* (=$\sqrt{6{D}_{0}{\tau }_{{\rm{eff}}}}$). This means that water molecules would need to be able to diffuse without barrier or hindrance for at least 40 *μm*. Assuming axons roughly 1 *μ*m in diameter (*d*), such a characteristic free displacement (*x*) would only occur with an axonal density of about 0.0005 (=$\tfrac{\pi {d}^{2}}{2\sqrt{3}{(d+x)}^{2}}$) and with nothing but free water between axons (in particular no microglial cells). Apart from CSF space and chronic axonal loss (wherein the inflammatory response has subsided), such an axonal density appears unlikely. At diffusion times commonly used in research on humans (as in many applications of the free-water imaging^27,29–32^), the so-called extracellular free-water fraction might actually be an imperfect proxy to the extra-axonal restricted diffusion.

In this study, the fact that when the fraction of extra-axonal restricted diffusion increases the diffusivity *d*_ear_ decreases (Fig. 3E,F) may represent a transition from a small residual environment of CSF (which is otherwise excluded from our region of interest) to a larger environment of microglial cells which restrict the diffusion of water molecules. In future work, combining a compartment with free isotropic diffusivity and one with limited isotropic diffusivity might separately identify the presence of CSF and atrophy on one hand and the presence of microgliosis and neuroinflammation on the other hand.

The other findings from the temporal evolution of DIAMOND parameters corroborate previous findings from DTI studies. The time course of the DIAMOND axial diffusivity is remarkably similar to that of the DTI axial diffusivity^17–21,33^. The time course for the radial diffusivity is similar to the one reported in previous studies^17–21,33^. Some works^17–20^ have reported an additional weak increase in radial diffusivity in the acute phase which was not observed in the present study. There are three possible explanations for this discrepancy. First, the lesion site used in experimental setups influences the time course of the Wallerian degeneration process: myelin clearance in the peripheral nervous system occurs much earlier than in the central nervous system^14^. While the optic nerve is considered part of the central nervous system (unlike all other cranial nerves), the dynamics of its Wallerian degeneration may resemble that of other cranial nerves rather than the slower dynamics observed in the rest of the central nervous system. This would explain the discrepancy with studies on the optic nerve^17,19^. Second, the type of lesion used to elicit Wallerian degeneration may affect its timing. While rhizotomy was used in the present study, ischaemia^17,19^ and contusions^18^ were used in others. Third, the radial diffusivity in studies where no other parameter was available may have confounded multiple microstructural changes that are independently captured by the fraction of extra-axonal restricted diffusion (*f*_ear_) in the present study. Supporting this claim is the fact that the dynamics of the radial diffusivity in two studies^18,20^ exhibits a two-stage increase similar to the dynamics of the extra-axonal restricted diffusion in the present study. Furthermore, in the study by Zhang *et al*.^20^, only the correlation between radial diffusivity and Luxol fast blue optical density at 30 days after injury is reported to be significant while no significant correlation is reported at 38 hours, 3 days, and 7 days. The authors acknowledged that the changes in radial diffusivity occurring in earlier stages might therefore be due to pathological processes other than myelin clearance. The discrepancy in the temporal evolution of the radial diffusivity therefore appears to be spurious and our findings in fascicular axial and radial diffusivities corroborate previous findings from DTI studies.

The present study has two main limitations. First, the fraction of extra-axonal restricted diffusion *f*_ear_ correlates with the morphometric aspects of reactive microglia (namely large ameboid microglial cells)—not its other functional aspects. Reactive microgliosis is itself a complex pathological process which involves microglial phenotypic changes, and production of cytokines and chemokines. A note of caution is therefore in order: While the fraction of extra-axonal diffusion (*f*_ear_) appears to be a DCI marker of reactive microglia, it is not sufficient to fully characterize reactive microgliosis. The latter depends on the microglial specific phenotype and pathological status. For instance, in glioma, the tumor environment leads to a change in microglial phenotype which is different from the inflammatory phenotype and microglia activated in that way does not release proinflammatory cytokines but present other transcriptional changes^8^. Tissue analysis (*e*.*g*., histology, immunohistochemistry, RT-qPCR, ELISA) thus remain of paramount importance if the goal is to more comprehensively characterize reactive microgliosis. The two techniques are therefore complementary. While DCI enables whole-brain/spinal cord *mapping* of reactive microgliosis (*i*.*e*., it indicates *where* reactive microglia occurs), tissue analyses enable detailed *characterization* of the reactive microgliosis in one specific area (*i*.*e*., they indicate *what* aspect of reactive microgliosis is possibly occurring). Future developments may explore the use of *f*_ear_ mapping to guide biopsy by informing the investigator of potential loci of interest.

Second, the absence of longitudinal histology (which can be achieved by sacrificing rats at different time points^20^) prevents the definite one-to-one association of DIAMOND parameters and pathological features during the course of Wallerian degeneration. The claims in this paper rather relied on two sources of evidence: (i) the empirical comparison of DIAMOND parameters and histology at the final time point (51 days post-injury), and (ii) the comparison of the time course of DIAMOND parameters with the known dynamics of Wallerian degeneration from the literature. Future work will investigate longitudinal histology with immunostaining and comparison with DIAMOND parameters to investigate whether the early increase in the fraction of extra-axonal restricted diffusion indeed represents early recruitment of microglial cells.

## Conclusion

This study investigated the use of DIAMOND, a diffusion compartment imaging (DCI) model, for the *in-vivo* mapping of reactive microglia. Findings from the temporal evolution of the DIAMOND parameters revealed that the fraction *f*_ear_ and diffusivity *d*_ear_ of the extra-axonal restricted compartment are compatible with the known dynamics of reactive microgliosis while the evolution of parameters of the axonal compartment replicates the wealth of DTI findings. Comparison with histology demonstrated a strong correlation between the fraction of extra-axonal restricted diffusion and microglial density. These results provide the first histological evidence that DCI is capable of mapping reactive microgliosis. They lay support for the use of DCI in studies investigating the pathogenesis of neurological and psychiatric disorders wherein neuroinflammation may play a role.

## Methods

### Animal model of spinal cord injury

Female Long Evans rats (Janvier, 180–200 g) were used. Two groups were defined: a control group (3 rats) and an injured group (4 rats). Both groups were anesthetized using a rodent anesthesia system (Equipement veterinaire Minerve, Esternay, France) with vaporized Isofurane (Isoba, Schering-Plough Animal Health, Merck Animal Health, Bomeer, Netherlands) and underwent laminectomy at L2–L3 to expose the spinal cord. The injured group then underwent left unilateral rhizotomy from L2 to L3 performed with a microciser.

The rhizotomy model chosen is a selective section of the dorsal and ventral rootlets with no injury to the spinal cord. Therefore the sectioned axons are clearly identified and the extension of the lesion is controlled, predictable and reproducible. In this work, we focus on the lesion extending rostrally along the ascending fibers of the gracile fasciculus. The absence of direct spinal cord injury precludes the formation of intra-spinal hematoma and cavities that can be highly variable in contusion and section models. Furthermore, hematomas and the subsequent blood remnant create long term artefacts and can be responsible for poor image quality in the vicinity of the lesion site. The spinal cord damage in total spinal transection is often too extensive to allow a precise identification of the lesioned axons and would have prevented the use of the contralateral side as a control.

Following rhizotomy, muscles were sutured together and the skin was sutured. Post-operative care included subcutaneous administration of Baytril Enrofloxacin (2.5 mg/kg, once a day for 2 weeks), buprenorphine (0.01 mg/kg, twice a day for 3 days), and lactate ringer solution (5 mL/100 g, once a day for 5 days). The protocols were approved by the ethical committee for animal care of the health science sector of the Université catholique de Louvain. All methods were performed in accordance with the relevant guidelines and regulations.

### *In-vivo* DWI

DWI were acquired in injured rats before and 4, 13, 37, and 51 days after surgery. In control rats, only the pre-surgical and the 51-day post-surgical acquisitions were performed. For each image acquisition, rats were anesthetized with an isofurane-air mixture (2.5% for induction and 1–1.5% for maintenance). Rats were then placed in a dorsal decubitus position on a custom-made bed. Respiratory rate and rectal temperature were continuously monitored with a physiological monitoring unit (SA Instruments, Model 1025, USA). The body temperature was maintained constant at 37 °C with a circulating warm-water pad.

A TriPilot sequence coupled with respiratory gating was acquired before DWI acquisition and the experimenter confirmed (and corrected if needed) adequate positioning of the rats. All acquisitions were carried out on an 11.7 Tesla Bruker BioSpec MRI (Bruker, Karlsruhe, Germany). The transmitter volume coil (diameter 72 mm) and the receptive surface coil (4-channel, 3 cm × 3 cm) were coupled for the acquisition covering the T12-L4 vertebral segments. The magnet was shimmed to adjust the homogeneity using quadratic adjustment. The multi-shell DWI acquisition sequence included 18 non-weighted DW images (which were averaged to create a *b*_0_ image) and 6 shells of 36 gradient directions each at b-values: 300, 700, 1500, 2800, 4500, 6000 s/mm^2^. The voxel resolution was 0.1 × 0.1 × 1 mm^3^. The other acquisition parameters were *T*_*E*_ = 23 ms, *δ* = 4.5 ms, and Δ = 12 ms. The orientations of diffusion vectors were maximally separated within and across shells using Caruyer’s method^34^. The duration of each acquisition for each rat was around 2.5 hours. Correction for animal motion and Eddy current was achieved by affine registration of each scalar DWI to the *b*_0_ image. To this end, images were resampled to a resolution of 0.05 × 0.05 × 0.06 mm^3^ to allow improved multi-scale pyramidal registration.

### DIAMOND model

DIAMOND considers the presence of different microstructural environments in voxels. It represents the DWI signal at the voxel level as a weighted sum of signals arising from each of them. The weights represent the contribution of each environment to the DWI signal. In this work we focus on imaging the rat spinal cord and use a two-compartment DIAMOND model with one isotropic restricted and one anisotropic compartment. The isotropic restricted compartment captures the signal arising from water molecules that do not show a preferential direction of diffusion. It is represented by a single diffusion coefficient *d*_ear_. Because the value of this coefficient is estimated from the data and may be much smaller than the diffusion of free water at 37 °C, the isotropic compartment aims at capturing the signal arising from the extra-axonal restricted diffusion (unlike isotropic free-water compartment which typically captures partial volumes of cerebrospinal fluid).

The anisotropic compartment is represented by a continuous statistical distribution of diffusion tensors with a mean tensor **D** and a heterogeneity parameter $\kappa$ which encodes how concentrated the distribution is. The mean tensor **D** is itself parameterized by a fascicular radial diffusivity *λ*_⊥_ and a fascicular axial diffusivity *λ*_‖_ which are akin to their widely-known DTI counterparts. The parameter $\kappa$ is also represented by the equivalent heterogeneity index ${\rm{Hei}}=\frac{2}{\pi }{\rm{atan}}\frac{1}{\kappa }$ which ranges from 0 to 1. It has been shown that incorporating the heterogeneity parameter better represents the DWI signal leading to more reliable values for the tensor **D**^10^. We let *f*_ear_ be the fraction of the DWI signal explained by the isotropic compartment so that 1 − *f*_ear_ is the contribution of the anisotropic compartment.

For a *b*-value *b* and a gradient direction *g*, the signal attenuation *S*/*S*_0_ modeled by DIAMOND reads:

$$S/{S}_{0}={f}_{{\rm{e}}{\rm{a}}{\rm{r}}}{e}^{-b{d}_{{\rm{e}}{\rm{a}}{\rm{r}}}}+(1-{f}_{{\rm{e}}{\rm{a}}{\rm{r}}}){(1+\frac{b{{\bf{g}}}^{T}{\bf{D}}{\bf{g}}}{\kappa })}^{\kappa }.$$

At high b-values and with gradient directions aligned with the mean axonal orientation, the signal attenuation is such that it falls below the noise level and brings no relevant information about the tissue microstructure. To filter out these DWI and stabilize the estimation of the DIAMOND parameters, a DTI model was first estimated to determine the mean axonal orientation of the spinal white matter. DWI acquired with both a b-value > 4500 s/mm^2^ and a gradient orientation at a angle <70° from the mean axonal orientation were filtered out. The parameters *f*_ear_, *d*_ear_, $\kappa$, and **D** were then estimated at every voxel from the input DWI data using the method described in^10^.

### Region of interest

We defined a region of interest (ROI) covering the T12 (rostral to the lesion over the course of axons) to L2 (at the superior border of the lesion site) levels of the gracile fasciculus as follows. The cerebrospinal fluid was identified and the spinal cord was manually segmented on the *b*_0_ image. The hypo-intense signal of the anterior spinal vein on *b*_0_ image and the high FA of the corticospinal tract on DTI were used as landmarks to manually segment the gracile fasciculus. Vertebral levels were identified on an anatomical T1-weighted image acquired within the same acquisition. The ROI did not include any voxels close to the cerebrospinal fluid. The result is an ROI volume of approximately 200,000 voxels with in-plane segmentation. The corresponding levels on histology were determined by direct comparison with an atlas^35^.

### Histology

Fifty-one days after surgery, all rats were euthanized and transcardially perfused successively with phosphate-buffered saline (PBS) and with 4% phosphate-buffered formaldehyde to fix the tissues. After the perfusion, the spinal cords were extracted and post-fixed in cold 4% buffered paraformaldehyde overnight. The following days, the tissues were successively transferred to 10%, 20%, and 30% sucrose/PBS (w/w) baths maintained at 4 °C for one night each. The spinal cord pieces were then frozen and stored at −80 °C, cryopreserved in optimum cutting temperature (OCT) compound, and sliced axially in 20 *μ*m-thick sections using a cryostat (Leica CM1850, Leica Microsystems, Wetzlar, Germany).

Sections were stained with Luxol Fast Blue (LFB) for myelin integrity assessment^18^ and counterstained with Cresyl Violet for the Nissl substance. Immunohistochemistry with the anti-panneurofilament SMI-312 (1/1000, Covance, Emeryville, CA) for neuronal cell bodies^17,19,20^ and Iba-1 in combination with a secondary immunoperoxidase stain (1:200; Vector Laboratories, Burlingame, CA) for reactive microglia^20^. The staining was performed with Diaminobenzidine (DAB) substrate (Sigma-Aldrich).

### Histological processing

LFB, SMI-312, and Iba-1 images were transformed to greyscale intensity values using the rgb2grey function of MATLAB 2015a (Mathworks, USA). The LFB intensity is referred to as the myelin intensity. To assess the fraction of the volume occupied by neurofilaments and reactive microglia, a Matlab routine borrowing ideas from Puigvert *et al*.^36^ and Phoulady *et al*.^37^ was developed as follows. A range filter with a radius of 5 pixels was first applied to the greyscale images to highlight areas with sharp contrast (as are the neurites) using the function rangefilt. Multi-level thresholding was then applied to the filtered image using the multithresh function with default parameters and with four levels^38^. Pixels with intensity values above the maximum level were considered part of the neurites (for SMI-312) and microglia (for Iba-1) while pixels with values below this threshold were assigned to the background. The ratio of the number of neurite-labeled (respectively microglia-labelled) pixels over the number of background pixels was defined as the neurite density (respectively microglial density). In each slice of the ROI, the mean myelin intensity, neurofilament density, and microglial density were computed for the ipsilateral and contralateral side in the injured group and for both sides simultaneously in the control group.

### Statistical analysis

Histological findings were compared between the control group and the ipsilateral and contralateral side of the injured group. Values from the intensity of LFB staining, from neurofilament density, and from microglial density were averaged on each side and in each slice within the gracile fasciculus so that one value was recorded for each side of each histological slice of each rat. For the control groups, both sides were averaged together.

To assess the temporal evolution of DIAMOND parameters, the values at all spinal levels rostral to the lesion within the gracile fasciculus were used. At each time point, the value between the contralateral and ipsilateral sides were statistically compared. Since comparisons were performed at 4 time points and for 5 parameters, a Bonferroni correction for multiple comparisons (with 20 comparisons) was applied to the *p*-values and rejection of the null hypothesis was based on the corrected *p*-values.

Finally, to compare microglial density from histology and *f*_ear_ from DIAMOND, the *f*_ear_ maps were first downsampled so that the number of DIAMOND slices equaled the number of histological slices. The values of microglial density and *f*_ear_ were averaged in each slice and on each side of the gracile fasciculus independently. The Pearson correlation coefficient between glial density and *f*_ear_ was then computed over all slices. Downsampling the *f*_ear_ maps was preferred over upsampling the histological values as the latter would artificially inflate the sample size leading to artificially low *p*-values.

All two-sample tests were two-sample *t*-tests and rejection of the null hypothesis was based on a threshold at $p < 0.05$.

## Data Availability

Data will be shared upon reasonable request from any qualified investigator. The software to estimate the parameters of a DIAMOND model from a set of DWI is freely available upon request on Bitbucket (https://bitbucket.org).
